The article "Improved Chaotic Algorithm-Based Optimization Technology of Architectural Engineering Drawing Parameters" was published in 2022. Journal: Comput Intell Neurosci.

# Improved Chaotic Algorithm-Based Optimization Technology of Architectural Engineering Drawing Parameters

**DOI:** 10.1155/2022/1827209

**Published:** 2022-08-28

**Authors:** Xiaoqiu Ma

**Affiliations:** Department of Basic Science, Jilin Jianzhu University, Changchun 130000, China

## Abstract

The traditional methods deal with large sample data sets of architectural engineering drawings and they have high time complexity and space complexity as well. Their searching time is long and sometimes the results are unsatisfactory. Therefore, this paper proposes an optimization method designed for architectural engineering drawing parameters to overcome the limitations of the traditional methods. It is based on the improved chaotic algorithm. The algorithm proposes the optimization model of architectural engineering drawing (AED) parameters in the first phase. In the second phase, an improved chaos algorithm is used to optimize the parameters of architectural engineering drawing, and the modeling strategy of visual parameter optimization environment is constructed. Finally, the visualization parameter optimization process of architectural engineering drawing is completed. Through experiments, it is evidently observed that the method presented in this paper can effectively reduce the optimization time, improve the lighting illumination of buildings, and improve the optimization precision of architectural engineering drawing parameters. The proposed method considers multiple parameters and it has greater application ability in the field of architectural designs.

## 1. Introduction

### 1.1. Background Study

In recent 20 years, the parametric design of building engineering has gradually become a new topic in the field of design. Parametric design transforms the concern of architectural design result into the concern of design process and control. Parametric design gets rid of the traditional modeling methods of sketch initiation or pattern reproduction, but controls the establishment of design schemes through the modeling and optimization of parametric models [1]. The process of parametric design can be divided into site investigation, form-finding, design evolution, structural system, and structural logic [2]. The parametric design process and scheme generation are characterized by complexity and nonlinearity. Parametric design focuses on the information carried by architectural elements and follows certain norms and rules to create architecture from the bottom up [3]. Parametric design techniques impart advantages for architecture design processes. Architects apply these methods in their creation of design suggesting solutions at an earlier stage of the process to speed up the design process and enhance the accuracy [4].

### 1.2. Existing Literature

In [4], the authors propose a process based on parametric design creation. It combines architectural design with parametric modeling methods. This makes the design objectives more comprehensive and also supports the designers in finding architectural solutions. In [5], the authors propose an optimization algorithm for architectural engineering drawing parameters based on Spark parallel SVM. The Spark cluster was used to broadcast the training set of architectural engineering drawing parameters to each Executor in the form of variables. The parameter optimization process of parallel SVM is carried out. Task parallelism is applied in order to speed up the optimization speed. In [6], the researchers put forward building cover day feed parameters based on the firefly algorithm of intelligent optimization method. It improves the HATA experience model covering the simulation of the building. It shows good processing precision. In [7], the authors propose an algorithm study based on the adaptive determination of DBSCAN algorithm parameters. It generates candidate EPS and other parameters using the distribution characteristics of the data set itself. The algorithm can realize the full automation of clustering process and can choose reasonable EPS and other parameters. It shows high clustering accuracy. In [8], the authors state that the parametric optimization of an architectural object is an important design task. They also state that improvement is needed in the area of quality of a design solution. Also, there is a need to take care of energy efficiency in design. The authors compare the calculated compactness ratios of the external envelope for different storeyed buildings. In [9], the authors describe different approaches for the parameterization in architecture. They also provide the comparison of these approaches. They map the design process to parametric data flow in each of the approaches. In [10], the authors propose two approaches for parametric design creation (1) Creating models in architectural design and (2) Using various tools of applied mathematics. They state that both the approaches need optimization for the purpose of modeling in architectural design. Authors use an interdisciplinary approach for identifying the role of optimization in architectural design.

### 1.3. Contributions of the Paper

From the existing literature, it can be concluded that though there is a lot of research in the field of Parameters Optimization Model for Architectural Engineering Drawing, they have the problem of poor prediction accuracy. Some of the methods show good accuracy but have high processing time. This paper proposes an optimization technique of architectural engineering drawing parameters based on an improved chaotic algorithm. Our aim is to design a Parameter Optimization Model for Architectural Engineering Drawing which is accurate and faster as compared to the previous methods.

### 1.4. The Major Highlights Are as Follows:

1. Proposing parametric optimization model which is novel in idea.
2. Visual parameter optimization condition design is presented.
3. Parameter optimization process is devised.
4. Proposing the optimization method of building engineering drawing parameters using an improved chaos algorithm.

The following sections explain the proposed work.

## 2. Construction of Parameters Optimization Model for Architectural Engineering Drawing

This is a three phase process in which, first of all, find a set of optimal parameter values. In the next phase, that is, visual parameter optimization condition design, parameters that satisfy the specific conditions are chosen. These conditions have been mentioned in detail in Section 2.2. In the final phase, Parameter optimization process is explained.

### 2.1. Parametric Optimization Model

Parametric optimization is to find a set of optimal parameter values *α∗* ∈ *α* in the feasible region of the design vector *α*=[*T*_1_, *T*_2_, *T*_3_, ..., *T*_*n*−1_, *T*_*n*_]^*T*^, so that the objective function *J*=*f*(*α∗*) takes the minimum (or maximum) value. For the parameter optimization problem [7], if the design variable *α* is a set of parameters, then the design problem in *r* dimensional space can be discussed as in equation (1).

(1) $$\begin{array}{c} \alpha \prime ={\left[T_{1},T_{2},T_{3},...,T_{r}\right]}^{T}. \end{array}$$

It is clear that at this point *α*′ is a fixed point in the Euclidean vector space *E*^*r*^ (design space) composed of *α*, which can be expressed as *α* ∈ *E*^*r*^. When the design variable is a parameter, the objective function can be described as in .

(2) $$\begin{array}{c} J=\;f\left(\alpha \right)=f\left(T_{1},T_{2},T_{3},...,T_{r}\right). \end{array}$$

According to equations (1) and (2), the general form of the parametric optimization mathematical model can be expressed by equation (3).

(3) $$\begin{array}{c} \underset{\alpha \in D}{\min}f\;\left(\alpha \right), \end{array}$$

where the objective function *f*(*α*) is a real-valued function, and *D* is the domain of *f*(*α*). Equation (3) can also be written in a more general form as the following:

(4) $$\begin{array}{c} \left\{\begin{array}{c} \underset{\alpha \in D}{\min}f\left(\alpha \right){}^{\prime }\\ s.t.\;d\left(\alpha \right)=0\\ h\left(\alpha \right)\leq 0, \end{array}\right., \end{array}$$

where *α*′=[*T*_1_, *T*_2_, *T*_3_, ..., *T*_*r*_]^*T*^ is an *r* dimensional design vector, *d*(*α*)=[*d*_1_(*α*), *d*_2_(*α*), ..., *d*_*p*_(*α*)]^*T*^ is a *p* dimensional equality constraint, and *h*(*α*)=[*h*_1_(*α*), *h*_2_(*α*), ..., *h*_*q*_(*α*)]^*T*^ is a *q* dimensional inequality constraint.

In equation (3), since the design variable is unconstrained to take all the values in the domain *D*, it belongs to the unconstrained extremum problem. In equation (4), *α* ∈ *D* is constrained by equations (5) and (6), that is,

(5) $$\begin{array}{c} d_{i}\left(\alpha \right)=0,i=1,2,..,p, \end{array}$$

(6) $$\begin{array}{c} h_{j}\left(\alpha \right)\leq 0,j=1,2,..,q. \end{array}$$

Therefore, equation (4) is the constraint extremum condition.

### 2.2. Visual Parameter Optimization Condition Design

For the optimization of visual parameters, the following conditions should be defined:

- One of the key problems in optimizing the visual parameters of the mathematical model and graphical transformation of the system is in what form the mathematical model can be graphically or visually transformed [11]. In fact, the equation constraint of optimization problems, such as differential equation, difference equation, transfer function, equation of state, and other forms, is visualized by graphical display technology according to the modular modeling idea.
- The feasible region is the set of points in the design space that satisfy all the constraints.
- Excitation function of the system includes instruction function and interference function. In order to facilitate the comparison of dynamic characteristics of the system, some typical signal functions are generally selected as instruction signals, such as step function, impulse function, and random signal [12, 13].
- For example, the initial time *t*_0_ of the end and terminal conditions, the terminal time *t*_*f*_, the initial state *x*(*t*_0_), and the terminal state *x*(*t*_*f*_) are either given or arbitrarily valued according to the task conditions.
- For visual parameter optimization problems, the objective function is generally shown in equation (2).

### 2.3. Parameter Optimization Process

After the designers analyze and calculate a variety of architectural form design schemes, the final form scheme is obtained. From the perspective of natural lighting and ventilation, the position and size of the internal atrium of the building are further optimized [14]. The actual parameter optimization problem is usually solved by numerical iteration method [15].

For general (multi-objective) optimization problems, the algorithm flow is as follows:

In the first step, initial design vector *α*_0_ was selected. In the second step, feasible direction *s*_0_ was found. In the third step, step size factor *l*_0_ is selected along the feasible direction, and the new design vector is obtained from *s*_0_ and *l*_0_ as the following equation (7).

(7) $$\begin{array}{c} \alpha_{1}=\alpha_{0}+l_{0}s_{0}. \end{array}$$

The fourth step is to find a new design direction *s*_1_ and step length *l*_1_ from *α*_1_. Iterate one step forward from point *α*_1_ to point *α*_2_, and so on, many iterations. The iteration form from step *k* to step (*k*+1) is shown in equation (8).

(8) $$\begin{array}{c} \alpha_{k+1}=\alpha_{k}+l_{k}\mathrm{S,} \end{array}$$

(9) $$\begin{array}{c} f\left(\alpha_{k+1}\right)<=f\left(\alpha_{k}\right),k=0,1,2,.... \end{array}$$

The fifth step is to check whether the preset accuracy is reached at each iteration step. If it is, the minimum point is considered to have been found; otherwise, the iterative calculation should be continued. In this paper, equation (9) is taken as the criterion for the termination of iteration as shown in equation (10)

(10) $$\begin{array}{c} \frac{\left\|\alpha_{k+1}-\alpha_{k}\right\|}{\left\|\alpha_{k}\right\|}\leq X, \end{array}$$

where *X* is the given precision.

## 3. Optimization Technology of Building Engineering Drawing Parameters Based on Improved Chaotic Optimization Algorithm

The parameter optimization technique is applied for engineering drawing parameters. The steps are as follows:

1. Proposing an Optimization method of building engineering drawing parameters
2. Identifying the modeling strategy of visual parameter optimization environment.
3. Proposing the visualization of parameter optimization process, that is, identifying the optimal parameters.
4. Applying the chaos algorithm for verifying the optimization effect of this method on the parameters of architectural engineering drawing
5. Comparing the results with existing algorithms like SPARK SVM, firefly algorithm, and DBSCAN algorithm

In the design of visual parameter optimization environment, the following is chosen.

### 3.1. Optimization Method of Building Engineering Drawing Parameters

Chaos is a common phenomenon existing in nonlinear systems, and its motion is characterized by ergodic, randomness, and regularity [15]. Logistic mapping is a successful example of chaos research in nonlinear equations. It was originally used to describe the generation change rule of insect numbers. Logistic mapping is shown in equation (11).

(11) $$\begin{array}{c} x_{n+1}=\mu x_{n}\left(1-x_{n}\right)\;n=0,1,2\ldots , \end{array}$$

where *μ* is the control parameter, and *n* is a normal number. When 3.544090 ≤ *μ* ≤ 4, a chaotic trajectory can be iterated from any initial value *x*_0_  ∈ (0,1), which is traversed within the range of (0,1). The chaos optimization algorithm takes advantage of this traversal feature, and the basic steps are as follows:

One, in formulas (1) and (13), vector *x*_*n*_ is, respectively, endowed with *m* initial values with slight differences (not 0.25, 0.5, and 0.75), and *m* is the number of parameters to be optimized. After *k* iterations, *m* different chaotic variables *x*_*i*_(*k*) *i*=1,2, ..., *m* can be obtained.

Two, by mapping the chaotic variable *x*_*i*_(*k*) to the search space of the optimization variable, *X*_*i*_(*k*) can be obtained:

(12) $$\begin{array}{c} X_{i}\left(k\right)=c_{i}+d_{i}x_{i}\left(k\right), \end{array}$$

where, *c*_*i*_ and *d*_*i*_ are constants related to the variable search space [*a*, *b*], *c*_*i*_ = *a*, *d*_*i*_ = *b* − *a*. For the first chaotic optimization search (rough search), the optimization index is min *f*(*X*_*i*_). Let *f∗* be the current optimal solution, and *X∗* be the corresponding parameter combination. *f*(*X*_*i*_(*k*)) < *f∗*, Substitute *X*_*i*_(*k*) into the calculation optimization index *f*(*X*_*i*_(*k*)) successively, *f*(*X*_*i*_(*k*)) < *f∗*, then equation (13) is obtained.

(13) $$\begin{array}{c} f*=f\left(X_{i}\left(k\right)\right),X*=X_{i}\left(k\right). \end{array}$$

Otherwise, *X*_*i*_(*k*) is discarded. Until *f∗* star stays the same for some number of steps.

For the second chaotic optimization search (fine search), according to equation (14), a new chaotic variable *X*_*i*_(*k*′) is generated, and *a*_*i*_ is the control variable less than 1.

(14) $$\begin{array}{c} X_{i}\left(k{}^{\prime }\right)=X_{i}^{*}+\alpha_{i}\left(x_{i}\left(k{}^{\prime }\right)-0.5\right). \end{array}$$

Three, put *X*_*i*_(*k*′) in order to calculate the optimization index *f*(*X*_*i*_(*k*′)). If *f*(*X*_*i*_(*k*′)) < *f∗*, then *X∗*=*X*_*i*_(*k*′), *f∗*=*f*(*X*_*i*_(*k*′)). Otherwise, give up *X*_*i*_(*k*′). Until *f∗* remains unchanged for several steps, the result is output.

### 3.2. Modeling Strategy of Visual Parameter Optimization Environment

In the design of visual parameter optimization environments, MATLAB 5.2 is utilized as the numerical calculation engine of optimization operation, and uses SIMuLink K 2.2 as the visual modeling support environment of nonlinear parameter optimization systems. The modeling idea is based on the separability of the system, that is, the large-scale system can be divided into several subsystems, and the subsystems can be decomposed into more primitive subsystems. Subsystem itself is defined as a visual component or module with independent operation function, which generally includes several input and output ports and is connected with each other through data flow channel; its function is to transform the incoming data or signal. The way to construct the visual optimization model is to establish the overall optimization simulation model by connecting the component models (submodels or modules) that constitute the system model. If the component model itself is constructed from a more primitive component model, it can form a hierarchical or hierarchical structure of the visual model. Therefore, the visual module (component) graphic modeling system based on SIMULINK is an important part of the advanced visual parameter optimization environment. It can provide users with a flexible, fast, and easy to expand high-level visual integrated information processing platform [16].

One, the graphical modeling components of SIMULINK are directly connected with each other, and the interfaces with the submodules of each layer of the model are retained in the visual environment.
Two, for the complex nonlinear parameter optimization model, the separation system technology is used to decompose the complex model into several subsystems at the next level according to the function. For the large subsystem, it can be further decomposed into subsystems at the next level. For this reason, the top-down hierarchical structure of simulation is established by analogy.
Three, it enhances the ability of human-computer interaction in the process of optimization, enables the user to pause or terminate the iteration at any time in the process of optimization, and reprocesses the data after optimization.
Four, it allows users to modify the hierarchical structure, parameters, and iteration initial values of the optimization model at any time, and allows users to run and test the subsystems of each layer, respectively, which is convenient for users to optimize and locate the errors of the subsystems of each layer.
Five, subsystem reuse technology allows users to design (subsystem) or document can be reused many times.
Six, users can customize, modify, or expand the optimization model library and algorithm library. The six considerations can ensure that the optimization system has clear structure, is easy to modify independently, is easy to debug and maintain, and has good scalability. The visual optimization environment is mainly composed of the following six parts through seamless links:
  - The model library provides a visual modeling platform and auxiliary graphic modeling tools through graphical mode. The model component is composed of model library function modules in SIMuLinK 2.2, which is used to complete the connection, conversion, calculation, and result output of system simulation optimization model.
  - By calling MATLAB optimization toolbox, the optimization algorithm library can provide users with a variety of optimization algorithms for solving such problems as parameter optimization, unconstrained optimization, quasi Newton realization, least square optimization, nonlinear least square realization, constrained optimization, SQP realization, and multi-objective optimization. The optimization algorithm can also be designed and developed by users themselves.
  - Model management optimization model management includes simulation layer management and application layer management. Simulation layer management is used to create, modify, open and access system models, and define and modify submodel blocks, including parameters, types, and attributes; application layer management is used to manage the files of the models according to the optimization tasks, M-file and MDL-file are used to share resources between models or platforms
  - Optimization database management takes MATLAB language as host language to help users manage, access, retrieve, and analyze the data in the optimization process. It can also dynamically analyze the optimization process, dynamically modify model parameters with optimization data, and compare the results of system optimization under different conditions.
  - The optimization environment settings are mainly used to set foreground, foreground and relation types (line type, line width, color, etc.) in the visual modeling area, as well as the running environment settings
  - The virtual oscilloscope technology is applied in real-time monitoring, which can monitor and analyze the waveform of any number of ports (input or output) of the optimization model at any stage and any moment of the optimization process.

### 3.3. Visualization of Parameter Optimization Process

As mentioned in Section 3.2, the modeling and simulation strategy of SIMuLinK can be adopted to establish the visual parameter optimization environment of general nonlinear system, and the basic optimization process is as follows:

The first step is to determine the design variables, objective functions, and constraints of the optimization mathematical model; The second step is to build a visual optimization simulation diagram or signal flow diagram based on the system mathematical model; The third step is to build the optimization simulation diagram from the SIMULINK model library by calling the basic module or model component in second steps; The fourth step is to write the optimization M-file, specify the optimization algorithm, and call the MATLAB optimization toolbox subroutine; In the fifth step, the optimization operation is performed, and the results of each iteration are visualized and stored in the optimization database; The sixth step is to find the optimal parameters of the system automatically; The seventh step is the post-processing of the experimental data.

Flowchart of parameter optimization in architectural engineering drawing has been shown in Figure 1.

According to the process mentioned in Section 3.3, the optimization of architectural engineering drawing parameters is realized, and the performance of the building is improved.

## 4. Experimental Results

In order to verify the optimization effect of this method on the parameters of architectural engineering drawing, the optimization algorithm of architectural engineering drawing parameters based on spark parallel SVM (reference [5] method), the intelligent optimization method of building coverage antenna parameters based on firefly algorithm (reference [6] method), the algorithm based on adaptive determination of DBSCAN algorithm parameters (reference [7] method), and the algorithm based on improved chaos algorithm are adopted The optimization method of architectural engineering drawing parameters (this method) carries out comparative experiments on the optimization precision of architectural engineering drawing parameters, architectural lighting, and optimization time of architectural engineering drawing parameters, and carries out experimental analysis.

After identifying the optimization effect of the proposed method on the parameters of architectural engineering drawing, the results are compared with the adopted algorithm, that is, chaos algorithm in terms of accuracy, architectural daylighting intensity, and time. It has been found that our proposed model outperforms as compared with the methods proposed in research [5–7].

The Comparison of different parameters has been explained in detail as follows:

### 4.1. Comparison of Parameter Optimization Accuracy in Architectural Engineering Drawing

In order to verify the optimization efficiency of architectural engineering drawing parameters, the methods of literature [5], literature [6], literature [7], and this paper (proposed method) are used to verify the optimization accuracy of architectural engineering drawing parameters, and the results are shown in Table 1. Comparison of optimization accuracy of architectural engineering drawing parameters has been shown in Table 1.

According to the analysis of Table 1, the optimization accuracy of architectural engineering drawing parameters is different under different methods. When the building area is 100 m^2^, the optimization precision of the method in reference [5] is 68%, the method in reference [6] is 58%, the method in reference [7] is 62%, and the method in this paper is 99.8%. When the building area is 600 m^2^, the optimization accuracy of the method in reference [5] is 74%, that in reference [6] is 65%, that in reference [7] is 65%, and that in this paper is 99.2%. The average values of the optimization accuracy of the parameters in the architectural engineering drawing of the methods of literature [5], literature [6], literature [7], and this paper are 69.1%, 65.2%, 65.7%, and 98.2%, respectively. This method always has the highest optimization accuracy of the parameters in the architectural engineering drawing, which shows that this method can realize the effective optimization of the parameters in the architectural engineering drawing.

### 4.2. Comparison of Architectural Daylighting

In order to verify the optimization effect of architectural engineering drawing parameters, the actual intensity of architectural lighting under the method of literature [5], literature [6], literature [7], and the method of this paper is compared, and the specific results are shown in Table 2. The architectural daylighting intensity under different methods has been shown in Table 2.

According to Table 2, the daylighting intensity of buildings is different under different methods. When the distance between the two sides of the building is 1 m, the daylighting intensity of reference [5] is 370 lux, the daylighting intensity of reference [6] is 287 lux, the daylighting intensity of reference [7] is 353 lux, and the daylighting intensity of the proposed method is 500 lux. When the distance between buildings increases to 10 m, the daylighting intensity of reference [5] is 7 lux, that of reference [6] is 9.4 lux, that of reference [7] is 87 lux, and that of proposed method is 321 lux. This method has higher building daylighting intensity, which shows that the building has higher building daylighting intensity and better daylighting effect.

### 4.3. Comparison of Optimization Time of Construction Engineering Drawing Parameters

In order to verify the optimization efficiency of architectural engineering drawing parameters, the methods of literature [5], literature [6], literature [7], and this paper are used to detect the optimization time of architectural engineering drawing parameters, and the results are shown in Figure 2.

Analysis of Figure 2 shows that the optimization time of construction engineering drawing parameters is different under different building areas. When the building area is 50 m^2^, the optimization time of the method in reference [5] is 24 s, that in reference [6] is 13 s, that in reference [7] is 5 s, and that in this paper is only 1s. When the building area is 400 m^2^, the optimization time of building engineering drawing parameters of reference [5] method is 27 s, the optimization time of building engineering drawing parameters of reference [6] method is 21 s, the optimization time of building engineering drawing parameters of reference [7] method is 30 s, and the optimization time of building engineering drawing parameters of the proposed method is only 5 S. When the building area is 600 m^2^, the optimization time of the method in reference [5] is 31 s, that in reference [6] is 43 S, that in reference [7] is 40 s, and that in this paper is only 8 s. This method has low optimization time and high optimization efficiency.

## 5. Conclusion

In this paper, an optimization method of construction engineering drawing parameters based on an improved chaos algorithm is proposed. The optimization model of construction engineering drawing parameters is constructed. The optimization process of construction engineering drawing parameters is designed. The optimization of construction engineering drawing parameters is realized by using an improved chaos algorithm. The modeling strategy of visual parameter optimization environment is constructed. After applying the proposed work to the existing data, it is concluded that proposed method always has the highest optimization accuracy of architectural engineering drawing parameters. The average optimization accuracy of architectural engineering drawing parameters of this method can reach 98.2%. This indicates the efficiency of proposed method in realizing the effective optimization of architectural engineering drawing parameters. Secondly, higher daylighting intensity and better daylighting effect in the buildings are achieved. The daylighting intensity of this method can reach 321 lux when the distance is 10 m. The proposed method shows low optimization time and high optimization efficiency. When the building area is 600 m2, the optimization time is only 8 s. It can be concluded that the proposed improved chaos algorithm outperforms the existing work in terms of accuracy, achieving higher daylighting intensity effect in the buildings as well as reduction in time.

## Figures and Tables

**Figure 1:** Flow chart of parameter optimization in architectural engineering drawing.

**Figure 2:** Comparison of optimization time of construction engineering drawing parameters.

**Table 1:** Comparison of optimization accuracy of architectural engineering drawing parameters.

Area of structure (m^2^)	Optimization precision of architectural engineering drawing parameters (%)			
	Method in literature [5]	Method in literature [6]	Method in literature [7]	Proposed method
50	67	45	65	99
100	68	58	62	99.8
150	65	65	75	95.8
200	58	68	65	99.6
250	53	65	73	97.4
300	63	56	65	97.8
350	68	66	68	98.9
400	72	66	70	97.3
450	78	76	57	98.4
500	74	65	59	97.8
550	73	68	64	95.4
600	74	65	65	99.2
650	79	71	67	99.5
700	76	79	65	98.4
Mean value	69.1	65.2	65.7	98.2

**Table 2:** Architectural daylighting intensity under different methods.

Distance in the building (m)	Daylighting intensity of buildings (lux)			
	Methods in literature [5]	Methods in literature [6]	Methods in literature [7]	Proposed method
1	370	287	353	500
2	230	221	330	487
3	120	112	310	476
4	90	92	276	468
5	50	68	254	456
6	32	45	214	439
7	27	28	187	410
8	12	23	165	387
9	9	12	128	362
10	7	9.4	87	321
11	5	6	33	286
12	3	3.5	26	265
13	2	1.5	21	253
14	1	0.7	8	220
15	0.5	0.6	5.2	165

## Data Availability

The data used to support the findings of this study are available from the author upon request (maxiaoqiu@jlju.edu.cn).
